The article "Correlation among genetic variations of c-MET in Chinese patients with non-small cell lung cancer" was published in 2017. Journal: Oncotarget.

# Correlation among genetic variations of c-MET in Chinese patients with non-small cell lung cancer

**DOI:** 10.18632/oncotarget.23474

**Published:** 2017-12-20

**Authors:** Jianchun Duan, Xiaodan Yang, Jun Zhao, Minglei Zhuo, Zhijie Wang, Tongtong An, Hua Bai, Jie Wang

**Affiliations:** ^1^ Department of Medical Oncology, Cancer Hospital Chinese Academy of Medical Sciences and Peking Union Medical College, Beijing, China; ^2^ Key Laboratory of Carcinogenesis and Translational Research, Ministry of Education, Department of Thoracic Medical Oncology, Beijing Cancer Hospital and Institute, Beijing, China

**Keywords:** non-small-cell lung cancer, c-MET, protein expression, copy number, mutation

## Abstract

**Background:**

The purpose of our research was to determine the correlation of amplification, protein expression and somatic mutation of c-MET in IIIb-IV stage NSCLC (Non-small cell lung cancer). We also explored correlation of c-MET variation with clinical outcome.

**Results:**

c-MET expression was observed in 28.6% (56/196) cases, and among those 13.8% (27/196) were shown to be FISH positive. Only 2.67% patients in this study carried the c-MET mutation. Cases with c-MET FISH positive were all IHC positive ,but in IHC positive cases, only half were FISH positive. Among patients with IHC^2+^ staining, 35.5% was FISH positive, while cases with IHC^3+^ staining,64% was FISH positive. Both protein expression and copy number of c-MET did not significantly correlate with clinical prognosis in these patients treated with EGFR-TKIs.

**Conclusions:**

IHC could be used as a preliminary screening method for c-MET copy number amplification and should be confirmed by FISH only in IHC positive case which facilitate selection of ALK or MET inhibitor therapy.

**Methods:**

c-MET gene copy number, protein expression and somatic mutation for exon 14 were detected by fluorescent- *In-Situ*-Hybridization (FISH), Immunohistochemistry (IHC), and Denaturing-High-Performance-Liquid-Chromatography (DHPLC), respectively, in 196 NSCLC patients. The relationship between c-MET abnormalities and clinical outcome of targeted therapy was analyzed by McNemar's test.

## INTRODUCTION

The *c-MET* gene locates on 7q21-31 and encodes a tyrosine kinase [1] Deregulation of HGF/c-MET signaling pathway due to mutation, amplification, overexpression, or activation has been observed in many types of cancers. Overexpression of c-MET was found in 25–75% lung cancer patients [2, 3], gene amplification has been observed in 5–22% [2–4],and mutations in about 5% of tumors [5, 6].

Studies in patients of NSCLC treated with EGFR-TKIs (epidermal growth factor receptor tyrosine kinase inhibitors), including Iressa or Tarceva, have shown that acquired resistance to EGFR-TKIs due to c-MET over-expression in approximately 20% population [7], which cause PI3K/Akt pathway activity. A lung cancer with c-MET amplification also demonstrated high sensitivity to crizotinib, a tyrosine kinase inhibitor targeting the anaplastic lymphoma kinase gene (ALK), suggesting cancers with increased c-MET levels may be sensitive to ALK inhibitors [8]. At present, ongoing phase I/II clinical trials are being carried out with c-MET inhibitors on patients with lung cancer [9, 10], and some of them have shown the effect of inhibiting tumor growth [11]. Although many therapies targeting c-MET are part of ongoing clinical trials, there is no general consensus on how c-MET status should be tested in lung cancer tissues or what the relationship is between the results obtained by FISH and IHC. Therefore, the variability of c-MET status trial results likely reflects variations in the methodology and the interpretation of the test results.

This study aims to explore relationship between protein expression, gene amplification and the presence of mutations using different, complementary methods. We also assessed whether c-MET variation detected by the three methods was related to prognosis in lung cancer patients.

## RESULTS

### c-MET protein expression

c-MET expression can be observed in the cytoplasm of lung cancer cells, and was detected in 56 cases. c-MET-scores,determined by immunohistochemical analysis indicated that 51.5% (101/196), 19.9% (39/196), 15.8% (31/196), and 12.8% (25/196) of the cases were scored as 0, 1+, 2+ and 3+, respectively (Figure 1).

**Figure 1:** Relationship between c-MET protein expression and *MET* gene copy number in lung adenocarcinoma by IHC and FISH (**A** and **B**) show IHC with moderate (IHC2+) and strong (IHC3+) staining,respectively. (**C**–**F**) show FISH positive and negative specimens that have been divided into two groups based on IHC analysis.

Immunohistochemical staining data was also used to evaluate 28 patients with two-site metachronous specimens, including those that underwent bronchoscopic biopsies twice (*n* = 6), specimens from bronchoscopic biopsy/pulmonary operations (*n* = 3), samples from patients with bronchoscopic biopsy/other organ metastasis (*n* = 5), specimens from pulmonary operations/bronchoscopic biopsies (*n* = 2), pulmonary operation specimen/other organ metastasis (*n* = 4), and patients with organ metastatasis/second organ metastasis (*n* = 8). Positive staining for c-MET was detected in 17.8% (5/28) of first-site specimens and 25.0% (7/28) of re-biopsy samples . There were no significant changes observed between the two-site specimens in the majority of cases (*n* = 24). In total, four cases were positive (score 2+ and 3+) for both specimens, while in the twenty remaining cases, both two-site specimens were negative for c-MET staining (score 0) . Further, three cases changed from 0 to 3+ and one case went from strong (score 3+) to moderate (score 1+) staining when the first-site specimen was compared to the re-biopsy (Table 1).

**Table 1:** c-MET protein expression in patients with two-site tumors

IHC		First-site tumor		Total
		+	−	
Re-biopsy tumor	+	4	3	7
	−	1	20	21
		5	23	28

*P* = 0.002 *kappa* = 0.579.

### Evaluation of c-MET gene copy number by FISH

c-MET copy number was found to be positive by FISH in 13.8% cases (27/196), and the FISH patterns are illustrated in Figure 1. Using FISH analysis 86.2%, (169/196) patients were found to be FISH negative, while high polysomy and amplification of the c-*MET* gene was detected in 9.7% (19/196) and 4.1% (8/196) of patients, respectively. Among eight of those displaying c-*MET* gene amplification, six had a low levels (gene-to-chromosome ratio ranging between 2.5 and 3.5), and two had high levels of amplification, with approximately 15 and 21 copies.

In first-site and rebiopsy specimens, 10.7% (3/28) and 17.9% (5/28) were shown to be FISH positive, respectively. Further, when two-sites specimens were examined, three cases were identified where both tumors were positive, while both specimens were negative in the other 23 patients. In two cases, high polysomy of the *MET* gene was detected in rebiopsy tumors, but not in first-site tumors where the concordant rate of copy number polysomy or amplification between the first-site tumors and rebiopsy tumors was 92.9% (26/28) (Table 2).

**Table 2:** c-MET copy number analysis in patients with two-site tumors

FISH		First-site tumor		Total
		+	−	
Second-site tumor	+	3	2	5
	−	0	23	23
		3	25	28

*P* = 0.000 *kappa* = 1.000.

### c-MET gene mutation

One handerd and fifty paraffin-embedded tumor samples were available for gene mutation analysis. Four samples were found to harbor mutations. All mutations were localized in the intronic region upstream of the 5′splice site of exon 14. One of the identified mutations resulted in a 10-base deletion and the other three cases were single base substitution. All the four cases did not carry c-MET expression and copy number amplification.

### Association between protein expression and GCN of c-MET

In order to determine whether genomic DNA copy number variations contribute to gene expression changes, the correlation between *MET* gene expression and corresponding DNA copy number changes was determined (Table 3).

**Table 3:** Associations between protein expression and copy number in 196 pts

Item		FISH		Total
		FISH+	FISH–	
**IHC**	Negative	140	0	140
	Positive	29	27	56
		169	27	196

Overexpression of MET protein in tumor tissue relative to adjacent normal tissues occurs in 25–75% of NSCLC and is associated with poor prognosis.

*P* < 0.001, McNemar's test.

A positive correlation between high protein expression and increased copy number was identified and the consistency of two methods was 85.2% (167/196) (*P* < 0.001).Among 196 patients, 140 were both negative in IHC and FISH; 27 patients showed both positive in IHC and FISH. Twenty-nine cases showed positive only in IHC. Of 56 patients shown to be IHC positive, 27 were FISH positive. Conversely, patients with IHC negative were all FISH negative. The sensitivity and specificity of MET IHC analyses were determined to be 100% and 82.8%, respectively. In patients that were found to have no (score *=* 0, *n* = 124) or very faint (score *=* 1+, *n* = 16) MET staining, 22 cases were triploid and 4 were tetraploid for MET, respectively. Among those with moderate MET IHC staining ( score= 2+, *n* = 31), 11 (35.5%) of the tissues were FISH positive, including 9 (29.0%) with high polysomy and 2 (6.5%) with amplification of the *MET* gene. Among patients with high IHC staining (score *=* 3+, *n* = 25), 16 (64.0%) were determined to be FISH positive, including 10 (40.0%) with high polysomy and 6 (24.0%) with amplification (Table 4, Figure 1).There were significant differences between IHC intensity and FISH scoring (*p=* 0.034). Our data suggested that a low number of *MET* gene copies per cell had not influenced the level of protein expression, whereas cells with increased copy number, including those with high polysomy and amplification, had an impact on protein level.

**Table 4:** Association between protein expression and copy number in IHC positive pts

Item		FISH			Total
		FISH-Num (%)	High polysomy Num (%)	Amplification Num (%)	
**IHC**	2+,Num(%) 3+,Num(%)	20 (64.5) 9 (36.0)	9 (29.0) 10 (40.0)	2 (6.5) 6 (24.0)	31 25
**Total**		**29 (51.8)**	**19 (33.9)**	**8 (14.3)**	**56**

Overexpression of MET protein in tumor tissue relative to adjacent normal tissues occurs in 25–75% of NSCLC and is associated with poor prognosis.

*P* = 0.034, McNemar's test.

Interestingly, no changes were identified between first-site and re-biopsy samples with respect to MET overexpression or copy number in the majority of paired two-site cases. Only four changes were observed by IHC and two changes by FISH detection. There were three changes from scores of 0 to 2+ or 3+, which were confirmed in two patients by FISH. These was another single case where the IHC score went from 3+ to 0, when the first-site tumors were compared to the rebiopsy tumors. Further, four cases were identified with protein expression positive in both two-site tumors, and three of these were also found to be positive FISH analysis. In total, 20 patients showed protein expression both negative in two-site tumors by IHC and FISH both negative in 23 patients (Tables 1, 2). The distribution of FISH and IHC patterns, according to various clinicopathological parameters, is summarized in Table 6. There were no significant associations between the expression levels, GCN, and other clinicopathological variables.

**Table 5:** Association between clinical response to EGFR-TKIs and EGFR mutation/c-MET copy number

		EGFR-TKIs		
Item	Number of patients	PR	SD	response PD
**EGFR^mut^/MET^amp^**	5	2	2	1
**EGFR^mut^/MET^wild^**	39	14	22	3
**EGFR^wild^/MET^amp^**	1	0	0	1
**EGFR^wild^/MET^wild^**	13	0	3	10
**Total**	**58**	**16**	**27**	**15**

**Table 6:** Clinicopathological characteristics of patients and positive cases in FISH and IHC assay (*P* > 0.05)

Variables	Number	FISH Positive Num (%)	IHC Positive Num (%)
Age (mean ± sd,years)	57.5 ± 5.6		
Gender			
Female	97	12 (12.4)	26 (26.8)
Male	99	15 (15.2)	30 (30.3)
Smoking history			
Never	124	16 (12.9)	32 (25.8)
Former or current	72	11 (15.3)	24 (33.3)
Histologic type			
Adenocarcinoma	180	26 (14.4)	53 (29.4)
Non-ade	16	1 (6.3)	3 (18.8)
TNM stage			
I + IIIa	21	3 (14.3)	7 (33.3)
IIIb + IV	175	24 (13.7)	49 (28.0)

Overexpression of MET protein in tumor tissue relative to adjacent normal tissues occurs in 25–75% of NSCLC and is associated with poor prognosis.

### Prediction implications of c-MET protein expression and GCN

58 patients were treated with Gefitinib or Erlotinib orally once per day. Treatment was discontinued when the disease progressed or intolerable toxicities appeared.

Neither the overall response rate (ORR) nor progression free survival (PFS, Figure 2) in the different categories of MET protein expression or GCN showed significant differences.

**Figure 2:** Progression-free survival (PFS) curves for the 58 patients treated with Gefitinib or Elorinib (**A**) PFS curve by c-MET copy number measured by FISH. (**B**) PFS by c-MET protein expression measured by IHC. (**C**) PFS by EGFR mutation status.

As a correlative study, *MET* copy number analysis and the presence of the EGFR mutation were determined in these 58 tumor samples. Among these patients, 44 were found to be EGFR mutants (EGFR^mut^), and among them, 5 patients were also positive for *MET* amplification (EGFR^mut^/MET^amp^). Additionally, 14 cases were shown to be wild-type for EGFR (EGFR^wild^), with one patient also displaying *MET* amplification (EGFR^wild^/MET^amp^). Using the Response Evaluation Criteria in Solid Tumors, we determined that 16 (27.6%) patients achieved a partial response (PR), with a PFS of 19.23 months and 27(46.6%) achieved a stable disease (SD), with a PFS of 14.06 months, 15 (25.8%) showed progressive disease(PD), with a PFS of 1.70 months. The detailed information of clinical response and EGFR/c-MET variation was showed in Table 5.

Six patients received Crizotinib as a first-line or second/third-line therapy. Among these cases, ALK protein expression (Ventana IHC assay) was positive in three (ALK^pos^), MET was positive in one (MET^pos^), and ROS1 was positive in the remaining two (ROS1^pos^). The response to Crizotinib in the three ALK^pos^ patients were PR, while the single MET^pos^ patient showed SD, and both ROS1^pos^ patients both were found to have PD.

## DISCUSSION

The need for accurate detection of MET alteration has become much more important, from both a clinical and a molecular standpoint, because the subset of patients with NSCLC who will benefit from MET inhibition therapy are dependent on this information. MET amplification has also been accepted as one of the mechanisms of acquired resistance to EGFR-TKIs [12]. IHC and FISH are standardized methods for detecting protein expression and copy number in clinical practice, and results from these detection were important for clinical advantage patients screening. IHC could be as initially screening method due to its rapid and inexpensive advantage. Those with moderate or intense staining indicative of c-MET gene expression are then tested by FISH for confirmation of c-MET positivity because it is golden-standardized for copy number detection.

Previous studies describe much variation in the frequencies of MET protein overexpression (25–75%) and copy number variation (3.8–21%) in lung cancer [13–16], largely due to the use of different methods and specimens obtained in primary site or metastatic tumors. In the present study, we performed a direct comparison of *MET* GCN per cell using FISH with MET protein expression evaluated by IHC in therapy-naïve NSCLC. These data suggest that there is a significant correlation between increased GCN and high levels of MET protein expression. In this study, IHC and FISH positivity were found to be 28.6% and 13.8%, respectively.Detailed analyzing, we found patients with IHC score3+, 64% showed FISH positive, if patients with IHC score2+, only 35.5% showed FISH positive. Dziadziuszko *et al.* [4] performed the representative study on the correlation between MET protein accumulation and gene copy number. Their study included primary tumors from 189 surgically resected NSCLC patients, and showed that MET protein expression was positive in 25% by IHC, and copy number amplification or high polysomy was identified in 12.1% by SISH (Silver *in situ* hybridization). Our study showed similar results, with the exception that our cohort was comprised of advanced patients and the detection method used to measure copy number was FISH. All patients who displayed amplification (clusters) or high polysomy of the *MET* gene also were positive for MET protein expression, while only half of the IHC positive patients had amplification or high polysomy. These data suggest that IHC can be a viable, alternative screening method, subjected to confirmatory testing by FISH in IHC positive cases, for anti-MET therapy or monitoring of EGFR-TKIs acquired resistance. While patients with no IHC positive staining, indicative of altered *MET* gene expression, are considered FISH negative and therefore do not require reevaluation. However, a portion of lung carcinomas showed disomy while overexpressing the MET protein, suggesting that MET protein expression might also be controlled by mechanisms other than gene copy increase, including hypoxia-induced overexpression [17] and activated ERK/AKT induced MET overexpression through transcriptional mechanisms.

In our cohort, 28 patients had two-site tumors, which were obtained at diagnosis and during target therapy or chemotherapy. Among them, three patients changed from negative to positive of c-MET protein expression, and were all patients that received Tarceva as a first-line treatment. Further, they also received second biopsies to evaluate disease progression, which were confirmed by FISH in two patients that showed c-MET GCN gains involved in resistance to Tarceva. When EGFR mutation analysis was combined with MET copy number determination, the five patients with double mutations (EGFR^mut^/MET^amp^) showed PR and SD in four, while only one showed PD and was due to the T790M mutation. Our study suggested that although c-MET amplification preexists in some tumors, EGFR mutation was still most strongest predictor for EGFR-TKIs (Figure 2C). For the six patients that received Crizotinib, ALK expression was the best factor for predicting response, rather than MET protein expression or ROS1 translocation

In conclusion, our study provides detailed descriptive analysis of the relationship between *MET* gene copy number and MET protein expression using different comparisons, demonstrating a good association between these two markers. As MET inhibitors enter the clinical arena in the near future, our results suggest IHC could be as fast and reliable screening method which only should be confirmed by FISH in IHC positive patients.

## METHODS

### Patients and specimens

Formalin-Fixed-Paraffin-Embedded (FFPE) tissues from 196 NSCLC patients were obtained from the Tissue Bank of Thoracic Medical Oncology Department of Peking Cancer Hospital from 2012 to 2014. Ethics Committee of Peking Cancer Hospital had approved our research (approval number 2015KT09) and patients had written consent before recruited. The median follow-up was 19.7 (range, 8.7–34.2) months. Patient characteristics are summarized in Table 6.

Six patients received Crizotinib 250 mg twice daily until disease progression.

Among these patients, 28 had two-site metachronous specimens, including those from two bronchoscopic biopsies, bronchoscopic biopsy/pulmonary operations, and bronchoscopic biopsy/other organ metastasis, which was described in detail in the results section. The rebiopsy specimens were obtained after chemotherapy or target therapy for the purpose of surgery, identifying whether occurring pathological transformation or biomarker detection.

Fifty-eight patients received Gefitinib or Elortinib as first-line (*n* = 35) or above first-line treatment (*n* = 23) and EGFR gene mutation status was obtained by routine analysis.

### Immunohistochemistry (IHC)

All slides were processed under identical conditions using standard protocols. The antibody was diluted at 1:150 (Met (D1C2) XP^®^ Rabbit mAb ,Cell Signaling Technology, USA) using SignalStain antibody diluent (Cell Signaling Technology, USA), was applied to slides for 16 h at 4°C. Goat anti-rabbit secondary antibody (DAKO) was incubated for 15 min and then following by the routine staining procedure. The IHC score was classified as 0 to 3+according to staining strength in membrane: no staining or <10% tumor cells (score 0), faint staining in >10% (score 1+), moderate staining in >10% (score 2+), and strong staining in >10% (score 3+). Score 0/1+ and 2+/3+ were regarded as negative and positive respectively.

### Fluorescent *In Situ* Hybridization (FISH)

c-MET gene copy number (GCN) were carried out to validate the results of the immunohistochemical analyses. A commercially available probe cocktail comprised of green fluorochrome-labelled CEN 7 and Texas Red fluorochrome-labelled c-MET probe was used (Abnova, Taiwan). 100 cells in each section were analyzed according to the manufacturer's instructions. In Several criteria were used to asses c-MET gene status. A specimen was considered as c-MET amplification if any of the following conditions are met: (i) ≥10% of tumor cells showed ≥15 c-MET signals; (ii) tight c-MET signal clusters; (iii) signals of c-MET/CEN7 ratio >2. ≥50% of tumor cells containing more than five c-MET signals was considered as high polysomy . Samples that were considered both high polysomy and c-MET amplification were marked as FISH positive. Results of c-MET FISH and IHC were evaluated by two independent pathologists.

### c-MET and EGFR mutation analysis

For c-MET mutational analysis, the coding region of tyrosine kinase domain exon 14 was amplified from FFPE tissue DNA and analyzed by DHPLC and these positive samples were further verified by sanger sequencing. DHPLC analysis run on Transgenomic Wave Nucleic Acid Fragment Analysis System according to the manufacturer's protocol.

The primer for 5′ splice site of exon 14 were forward:5′- TATGTAGTCCATAAAACCCATGAG, reverse:5′- CTTACAAGCCTATCCAAATGAG.

The primer for 3′ splice site of exon 14 were forward: 5′-AAGTGTAAGCCCAACTACAGAA, reverse: 5′- GAGGTAAATACTTCCTTTAGGTTT.

AmoyDx^TM^ EGFR 29 Mutations Detection Kit (Amoy Diagnostics Co, XiaMen, China) was used for EGFR mutation detection.

### Statistical analysis

Comparative analysis of IHC and FISH was used McNemar test . The correlation of variables were analyzed by chi-square test and if value < 5, Fisher's exact test was used. The log-rank test was used to analyzed relationship between each group and survival. Statistically significant was set as *P* < 0.05. All calculations were performed by SAS (SAS Institute, Inc., Cary, NC).

## Abbreviations

NSCLC: Non-Small-Cell Lung Cancer
GCN: gene copy number
IHC: Immunohistochemistry
FISH: fluorescent In Situ Hybridization
DHPLC: Denaturing High Performance Liquid Chromatography
